The article "Effects of Acupuncture Combined with Biofeedback Therapy on Limb Motor Rehabilitation in Patients with Acute Stroke: Systematic Review and Meta-Analysis" was retracted in 2023. Reasons: signs of a paper mill; compromised peer review; unreliable results or conclusions.

# Effects of Acupuncture Combined with Biofeedback Therapy on Limb Motor Rehabilitation in Patients with Acute Stroke: Systematic Review and Meta-Analysis

**DOI:** 10.1155/2022/9582077

**Published:** 2022-07-05

**Authors:** Xinrong Song, Xiaoge Zhang, Yan Weng, Yu Liu, Qi Shan, Wenna Chen, Wanwan Ma, Qi Dong, Dandan Qu, Yibo Guo, Jie Xiong, Fuhua Deng, Qizhi Fu, Yufu Xin

**Affiliations:** ^1^The First Affiliated Hospital and College of Clinical Medicine of Henan University of Science and Technology, Luoyang 471003, China; ^2^Department of Rehabilitation, The First Affiliated Hospital of Henan University of Science and Technology, Luoyang 471003, China; ^3^Department of Intensive Care Unit(Internal Medicine), The First Affiliated Hospital, And College of Clinical Medicine of Henan University of Science and Technology, Luoyang 471003, China; ^4^Department of Intensive Care Unit, Songxian People's Hospital, Luoyang 471400, China; ^5^Department of Neurology, The Second Affiliated Hospital of Henan University of Science and Technology, Luoyang 471003, China; ^6^Harbin Medical University, Pharmacy College, Harbin, Heilongjiang 150081, China

## Abstract

**Objective:**

The purpose of the systematic review is to verify the effect of biofeedback therapy on limb motor rehabilitation in patients with acute stroke and to provide evidence-based medicine for the promotion and use of biofeedback therapy.

**Methods:**

The randomized controlled trials (RCT) of biofeedback therapy in the treatment of cerebral palsy were searched in PubMed, EMBASE, ScienceDirect, Cochrane Library, China National Knowledge Infrastructure (CNKI), China VIP Database, Wanfang Database, and Chinese Biomedical Literature Database (CBM). The starting time and ending time of this study are from the time of building the database of the number of pieces to October 31, 2018. The data included in this study were extracted by two independent researchers and evaluated the bias risk of all the literature included in the study according to the Cochrane manual 5.1.0 criteria. RevMan5.4 statistical software was used to analyze the collected data by meta.

**Results:**

This systematic review included 9 RCT studies with a total of 1410 patients. The results of meta-analysis showed that there were significant differences in the improvement of lower limb muscle tension, comprehensive spasm scale score, EMG score, and passive range of motion of ankle joint between biofeedback therapy and routine rehabilitation therapy.

**Conclusion:**

Biofeedback therapy can improve lower limb muscle tension, spasticity, EMG integral value, and passive range of motion of ankle joint in children with cerebral palsy and provide better conditions for improving the motor ability of lower extremities in children with cerebral palsy. However, more studies and follow-up with higher methodological quality and longer intervention time are needed to further verify.

## 1. Introduction

Stroke is a group of diseases in which brain tissue is damaged due to sudden rupture of blood vessels in the brain or blockage of blood vessels resulting in blood circulation disorders. Most of them appear in the form of hemiplegia, commonly known as “hemiplegia.” China is one of the countries and regions with a high incidence of stroke. According to epidemiological estimates, the annual incidence of stroke in China is about 150/100000 and 70%–80% of the survivors have motor dysfunction. The form of “hemiplegic” is the most common [1]. Hemiplegia is a disease of the central system, whose pathological mechanism is pyramidal tract injury, which leads to central paralysis. In clinic, it can be manifested as the flexor model with upper limb symptoms and the extensor model with lower limb symptoms. Hemiplegic patients with stroke basically lose the ability to live independently, which undoubtedly increases the burden on the family and society but also causes harm to the physiology and psychology of the patients. With the continuous progress of modern medicine and the development of medical technology, the mortality rate after stroke has been significantly reduced but the disability rate is as high as 70% and 80% [2]. Trauma, cerebrovascular accident, burn, and peripheral nerve injury can impair hand function in varying degrees, and stroke is one of the main causes of serious hand dysfunction [3]. According to the principle of neurodevelopment, the functional recovery of lower limbs after stroke is faster than that of upper limbs and the recovery of the proximal limb is faster than that of the distal limb. Therefore, the recovery of hand function of hemiplegic patients is longer than that of other limb disorders [4]. In addition, due to the fine and complex anatomical structure of the hand, the recovery of hand function after hemiplegia is more difficult than that of other limb functions. It is reported that about 80% to 90% of poststroke hemiplegic patients have a certain degree of spasm [5]. Hand spasm in hemiplegic patients after stroke is a manifestation of abnormal muscle tone after upper motor neuron injury, which is caused by increased activity of spinal cord reflex and is characterized by the increase of stretch reflex with the increase of speed. It is caused by the loss of regulation of stretch reflex in the higher center after stroke [6]. In short, the recovery of hand dysfunction is difficult and time-consuming, which is not only a difficult problem for rehabilitation workers, but also brings many difficulties and challenges to the rehabilitation training of the upper limb and hand function of hemiplegic patients because of hand spasm. Therefore, the research on time saving, labor reduction, efficient hand function rehabilitation equipment, and rehabilitation training model has become the research focus of stroke hemiplegia [7]. Therefore, more and more attention has been paid to the rehabilitation of hemiplegic patients with stroke. Acupuncture has the function of holistic and two-way regulation, and its low cost and little side effects play a special role in the recovery of motor function of hemiplegic patients [8, 9].

At present, there are many methods for the treatment of stroke, such as selective posterior rhizotomy, exercise therapy such as Bobath and Vojta, use of gangliosides and other nutritious brain nerve drugs, acupuncture, and other traditional Chinese therapy. Surgery is one of the effective methods for the treatment of hemiplegia, but it also has some disadvantages, such as improper operation, lack of experience, or other uncontrollable factors. Therefore, in addition to the operation, it is particularly important to find a new noninvasive treatment. However, because stroke has three stages: acute stage, recovery stage, and sequela stage, the effect of acupuncture single therapy on improving lower limb motor function of hemiplegic patients is not obvious. If TCM acupuncture and moxibustion can be combined with rehabilitation medicine theory, acupuncture combined with rehabilitation training will play an important role in the recovery of lower limb motor function in hemiplegic patients with stroke. Biofeedback therapy takes the weak electrical signal of muscle spontaneous contraction as the signal source and turns it into visual signal, and the whole training process is closer to the game, so that the children can train actively through systematic hints and doctor guidance and learn to control their own movements [10]. Puf et al. [11, 12] show that EMG biofeedback therapy can inhibit the muscle tension of spasmodic muscles. Cevolani et al. [13] focused on biofeedback therapy to improve ankle function in children with cerebral palsy. Ansell and Huizenga et al. [14, 15] and other scholars gradually applied biofeedback therapy to improve walking function in children with cerebral palsy. Wu et al. and Bae et al. [16, 17] believe that biofeedback therapy can effectively improve ankle strength (37.7%), knee extension angle (7.4°), and step size (12.7%). Functional gait training can increase patient participation and magnify the effect. A large number of literatures have shown that biofeedback therapy is used in the clinical treatment of lower limb motor function in stroke but there is no systematic evaluation of the efficacy of spasm. Therefore, the purpose of this study is to systematically evaluate the effect of acupuncture combined with biofeedback therapy on limb motor rehabilitation in patients with acute stroke through the method of meta-analysis, so as to provide reference basis for the application and promotion of biofeedback therapy in clinical rehabilitation.

## 2. Research Contents and Methods

### 2.1. The Sources and Retrieval Methods of Documents

The Chinese Journal full-text Database (CNKI), VIP full-text Database (VIP), Wanfang Database, and Chinese Biomedical Literature data (CBM) were searched by computer, and the relevant Chinese journals, conference papers, and degree papers were searched. With the method of literature review, the data about the recovery effect of lower limb motor function in Chinese patients with hemiplegia in the early stage of stroke were collected. Literature retrieval was conducted in the form of free words and subject words, with the key words of acupuncture, rehabilitation training, stroke hemiplegia, motor function, etc. The starting time and ending time of this study are from the time of building the database of the number of pieces to October 31, 2018. The data included in this study were extracted by two independent researchers and evaluated the bias risk of all the literature included in the study according to the Cochrane manual 5.1.0 criteria.

### 2.2. Literature Inclusion Criteria and Exclusion Criteria

#### 2.2.1. Literature Inclusion Criteria

*(1) Study Type*. All hemiplegic patients with stroke in China were treated with acupuncture combined with rehabilitation training and routine treatment (RCT). The language was limited to Chinese.

*(2) Subjects*. Patients with hemiplegia after stroke (cerebral infarction or cerebral hemorrhage) met the diagnostic criteria of stroke revised by the fourth National Cerebrovascular Academic Conference in 1996 by clinical diagnosis and CT or MRI examination, and patients with lower limb dysfunction caused by mental disorders and skeletal muscle diseases were excluded.

*(3) Intervention*. The patients in the control group were treated with routine treatment, and the patients in the experimental group were treated with rehabilitation training combined with acupuncture: (1) routine treatment: routine therapy (drug therapy) in the department of neurology; (2) rehabilitation training: (a) active training, which mainly includes turnover training, sitting training, transfer training, and walking training, the purpose of which is to prevent muscular dystrophy; (b) passive training, which mainly includes joint range of motion training and joint and abdominal muscle extrusion training, with the purpose of improving the joint range of motion; and (c) physical training, mainly using physiotherapy instruments to stimulate the lower limb nerves of stroke patients with hemiplegia, in order to promote the excitement of lower limb nerves, increase muscle tension, and improve their motor function; and (3) acupuncture therapy: including acupuncture treatment at Zusanli, Sanyinjiao, Neiguan, Hegu, and Taichong points.

#### 2.2.2. Literature Exclusion Standard

(1) It is not a randomized controlled study, (2) the data report is incomplete and the data cannot be used, (3) repeat the research content and take the latest research, and (4) the evaluation of the efficacy of the study is not limited to the recovery of lower limb motor function in stroke patients with hemiplegia

### 2.3. Outcome Index

The Fugl-Meyer motor function score includes the lower extremity score (FMA-L), walking function score (FCA), and lower extremity Brunnstorm stage score. A Fugl-Meyer score < 50 is classified as grade I, indicating severe dyskinesia; a Fugl-Meyer score of 50–84 is classified as grade II, indicating obvious dyskinesia; a Fugl-Meyer score between 85 and 95 is grade III, indicating moderate dyskinesia; a Fugl-Meyer score of grade IV between 96 and 100 indicates mild dyskinesia [18].

### 2.4. Quality Evaluation and Data Extraction

#### 2.4.1. Quality Evaluation

The quality of the included literature was evaluated by the Jadad scale, which was evaluated according to a random, blind method and loss of follow-up/withdrawal. 0-5 points were used to count. When the literature quality is less than 2 points, it is lower, and when it is ≥3 points, it is higher. The specific comments are as follows: (1) random: (a) 2 points: “random distribution” is mentioned in the literature and described in detail; (b) 1 score: “random distribution” is only mentioned in the literature but not explained; and (c) 0: the random allocation method/random allocation/pseudorandom allocation was not mentioned in the literature; (2) blind method: (a) 2 points: the “double-blind” method is used in the literature and the specific process is described correctly; (b) 1: the “double-blind” method is not specifically described in the literature; and (c) 0: no “double blind” method/method error; and (3) withdrawal/loss of follow-up: (a) 1: the number and reasons of withdrawal and loss of follow-up are described in detail in the literature and (b) 0: it is not mentioned in the literature.

#### 2.4.2. Data Extraction

Two evaluators independently extracted and crosschecked the literature. When the two people had differences, they reached an agreement through consultation. It includes the following: study author, publication time, sample size, treatment method, and curative effect evaluation method.

### 2.5. Statistical Processing

The RevMan5 software provided by the Cochrane collaboration network was used for meta-analysis. The mean and standard deviation of each Fugl-Meyer motor function score, walking function score, and net change difference of lower limb Brunnstrom staging index before and after intervention in the experimental group and the control group were input into RevMan5 for analysis. Because the index is a continuous variable, the weighted mean difference (WMD) is used as the effect scale, the 95% confidence interval was selected, and the *χ*^2^ test was used to determine whether there was heterogeneity among the studies. If *P* > 0.05 and *I*^2^ < 50%, the included studies were considered to be homogenous and a fixed effect model could be used for meta-analysis. If *P* < 0.05 and *I*^2^ ≥ 50% and the combined effect size is required to judge the homogeneity of the included studies, a random effect model will be selected. When the result of heterogeneity test is *P* < 0.05 and the source of heterogeneity cannot be determined, meta-analysis is considered to be inapplicable and the results should only be presented in the form of descriptive review.

## 3. Results and Analysis

### 3.1. The Results of Literature Retrieval and the Basic Situation of Literature Inclusion

452 articles were retrieved through the computer database, 269 articles were obtained after eliminating repeated studies, 161 articles were obtained by preliminary reading of the titles and abstracts, 23 articles were included after excluding irrelevant studies, reviews, case reports, and noncontrol literatures, then, 15 articles with incomplete data and no main outcome indicators were read carefully, and finally, 8 RCT articles were included. A total of 750 samples were analyzed by meta-analysis. The basic features included in the literature are shown in Table 1.

### 3.2. Evaluation of the Quality of the Methodology Included in the Literature

All the 8 RCT literatures included in this meta-analysis reported the baseline status of patients, only 2 RCT mentioned “random assignment” without any explanation, and the rest did not mention “random” information. The five studies included all gave detailed intervention measures and follow-up time. The number and reasons of the blind method and loss of follow-up or withdrawal were not described in detail in 8 RCT articles. According to the Jadad scale, it was found that all the 8 articles had RCT ≤ 2 points.

### 3.3. Meta Analysis Result

#### 3.3.1. Fugl-Meyer Motor Function Assessment Lower Limb Score

Through the inclusion of 8 RCT studies, with a total of 750 samples, the lower limb scores of Fugl-Meyer motor function evaluation between the experimental group and the control group were analyzed by meta-analysis. The results of the heterogeneity test showed that chi^2^ = 4.34, df = 4, *P* = 0.31 > 0.05, and *I*^2^ = 16%, indicating that there was no obvious heterogeneity among the included research data, and the combined effect of WMD was analyzed by the fixed effect model. The analysis of Figure 1 shows that the confidence interval of 95% of the combined effect of WMD was (5.77,6.15) and the test of the combined effect of WMD was Zhuan 62.24 (*P* < 0.00001). According to the results of this analysis, it can be considered that there is a statistical difference in the WMD of lower limb Fugl-Meyer motor function evaluation between the stroke hemiplegic patients treated with acupuncture combined with rehabilitation training and the stroke hemiplegic patients treated with routine treatment. The 95% confidence horizontal line of WMD falls on the right side of the invalid line, indicating that the lower limb score of Fugl-Meyer motor function evaluation of stroke hemiplegic patients treated with acupuncture combined with rehabilitation training is significantly higher than that of stroke hemiplegic patients treated with routine treatment.

#### 3.3.2. FCA Walking Function Score

Through the inclusion of 8 RCT studies, with a total of 750 samples, the FCA walking function score between the experimental group and the control group was analyzed by meta-analysis. The results of the heterogeneity test showed that chi^2^ = 2.39, df = 4, *P* = 0.66 > 0.05, and *I*^2^ = %, indicating that there was no heterogeneity among the included research data, and the combined effect WMD was analyzed by the fixed effect model. According to the analysis of Figure 2, the combined effect of WMD was 2.66, the confidence interval of 95% was (2.60,2.72), and the test of the combined effect dose WMD was *Z* = 82.12 (*P* < 0.00001); according to the results of this analysis, it can be considered that there is a statistical difference in the WMD of FCA walking function score between the stroke hemiplegic patients treated with acupuncture combined with rehabilitation training and the stroke hemiplegic patients treated with routine treatment and the 95% confidence line of WMD falls on the right side of the invalid line. The results showed that after acupuncture combined with rehabilitation training, the FCA walking function score of stroke hemiplegic patients was significantly higher than that of stroke hemiplegic patients treated with routine treatment (*P* < 0.05).

#### 3.3.3. Lower Limb Brunnstrom Staging Score

Through the inclusion of 8 RCT studies, with a total of 750 samples, the lower limb Brunnstrom staging scores between the experimental group and the control group were analyzed by meta-analysis. The results of the heterogeneity test showed that chi^2^ = 1035.42, df = 4, *P* < 0.00001, and *I*^2^ = 100%, indicating that there was obvious heterogeneity among the included research data, and the combined effect WMD was analyzed by the random effect model. According to the analysis of Figure 3, the combined effect of WMD was 1.06, the 95% confidence interval was (0.94,1.18), and the test of combined effect WMD was *Z* = 17.52 (*P* < 0.00001); according to the results of this analysis, it can be considered that compared with the stroke hemiplegia patients treated with acupuncture combined with rehabilitation training, the WMD of the lower extremity Brunnstrom staging score is statistically different and the 95% confidence level of the WMD falls below the horizontal line. On the right side of the ineffective line, it shows that the lower extremity Brunnstrom staging score of stroke hemiplegia patients treated with acupuncture therapy combined with rehabilitation training is significantly higher than the lower extremity Brunnstrom staging score of stroke hemiplegia patients treated with conventional treatment. Due to the small number of studies included in the analysis, it is not suitable for funnel plots but the analysis may have a certain degree of publication bias.

## 4. Discussion

Stroke, also known as stroke and cerebrovascular accident (CVA), is a group of cerebrovascular diseases characterized by sudden onset, rapid occurrence of local or diffuse brain function defects, and organic brain damage, including ischemic stroke and hemorrhagic stroke. The main clinical manifestations are hemiplegia, partial loss of sensation or even complete disappearance, dysarthria or even aphasia, dysphagia, and coma. Its morbidity, disability, and mortality are very high, and it is the most common cerebrovascular disease in the middle-aged and elderly population. Some data show that there is a trend of getting younger [19]. Clinically, it is not uncommon for patients in their thirties and forties to be young. According to the abstract [20] of the 2017 China Stroke Prevention and Treatment report, cardiovascular and cerebrovascular diseases were the world's leading cause of death in 2016, with more than 17.6 million deaths worldwide, including more than 5.5 million deaths caused by cerebrovascular diseases. Global epidemiological survey shows that the burden of stroke in China will continue to rise. Stroke is one of the three leading causes of death in the world. The third citizen death survey report released by China in 2008 showed that stroke had become the first cause of death (136.64/100000) [21]. According to statistics, the incidence of stroke in China is 120180/100000 and about 2 million new cases occur every year, of which about 80% are left with motor dysfunction of the lower extremities. Patients often show abnormal walking gait in the early stage of the disease [22]. Moreover, due to the decrease of muscle strength and muscle tension of the affected lower limbs, the active control ability of the patients is weakened, which seriously affects the motor function of the patients and leads to the decline of self-care ability. It brings heavy pressure and economic burden to the society and families. Therefore, at present, there is a major problem in the treatment of stroke, that is, the quality of life of hemiplegic patients after stroke. Hemiplegic patients after stroke generally have walking dysfunction and low self-care ability, so the current research hotspot and key point of neurology and rehabilitation department are to improve their self-care ability and improve their quality of life through the implementation of intervention measures. Return to society as much as possible. Clinical studies show that [23] more than 70% can restore walking ability through quasirehabilitation training, but because the development of stroke rehabilitation in China is relatively backward, most stroke hemiplegic patients do not receive formal rehabilitation treatment. The quality of life has been seriously affected. Patients with stroke often leave abnormal gait, and the weight-bearing and self-control abilities of the affected lower limbs are out of balance, which can increase the muscle tension of the lower limbs, resulting in pathological gait such as foot ptosis and foot varus [24]. Some patients use physiotherapists to assist the transfer of the affected side and center of gravity, but the treatment and repetition times are greatly limited due to objective reasons. At present, it is impossible for traditional physiotherapy to input tens of thousands of correct movements to patients, it is extremely difficult to correct the changes of patients' center of gravity and stride system, and it is difficult to achieve high-intensity and repetitive training requirements. The effect of gait recovery treatment for hemiplegic patients with stroke is limited. In the face of apoplectic hemiplegia, which is one of the four stubborn diseases of traditional Chinese medicine, although there are traditional Chinese medicine rehabilitation treatment methods such as traditional Chinese medicine decoction, acupuncture, massage, and scraping along meridians, the treatment cycle is long and the effect is not ideal [25].

The epidemiological situation of stroke in China and even the world is becoming more and more serious, and the responsibility of effective prevention and treatment of stroke is extremely urgent. In the clinical treatment and rehabilitation of stroke, rehabilitation training through clinical practice is the most effective way to improve poststroke dysfunction [26]. It can prevent complications such as joint stiffness, muscle spasm, and muscle atrophy, improve activities of daily living (ADL), reduce the burden of the family and society, and let patients return to their families and integrate into the society as soon as possible. According to modern rehabilitation medicine, stroke hemiplegia is that the higher center loses its ability to control arbitrary motor function, which is replaced by abnormal movement patterns under low central control [27]. Brunnstrom divided the recovery of motor function of hemiplegic patients into six stages: relaxation stage, muscle tone and combined exercise stage, muscle spasm stage, common movement and primitive posture reflex stage, separated movement stage, spasm basically disappeared stage, and coordinated movement basically normal stage [28]. The recovery of motor function of hemiplegic patients is actually to break the abnormal movement pattern under the low central control and establish a normal movement pattern in the later stage of recovery [29].

A large number of foreign studies have shown that acupuncture can improve the blood supply to the brain and promote the recovery of nerve cell function, while rehabilitation training can prevent and correct the emergence of hemiplegic spasm patterns such as joint contracture and limb stiffness [30]. Clinical practice has proved that acupuncture is an effective means for the treatment of cerebral stroke. Early acupuncture intervention can make use of vasodilation, promote blood circulation, reduce blood viscosity and platelet aggregation, improve blood microcirculation, improve the process of oxygen metabolism of brain cells, increase cerebral blood flow, and improve cerebral ischemia and hypoxia. Promote the establishment of collateral circulation of cerebral vessels. Activate the cerebral neural pathway [31]. There are many schemes for the treatment of stroke, one of the more classic schemes is to increase the energy supply of brain tissue; after mitochondria get enough nutrition, promote metabolism, which can protect central neurons, reduce lactic acid accumulation, and help to reduce the oxygen consumption rate. Reduce neuronal apoptosis. In addition, effective metabolism can reduce the content of fibrinogen and avoid the formation of cerebral thrombus [32]. Acupuncture treatment can dredge channels and collaterals, soften tendons to stop spasm, reconcile yin and yang, promote the relief of limb spasm in hemiplegic patients, and improve the function of fine movement of limbs: “where the twelve meridians are, the part of the skin. Therefore, at the beginning of all diseases, it must be prior to the fur.” It shows that the disease is first affected by the muscle surface of the body and the twelve meridians are closely related to the meridians and viscera. Acupuncture can effectively stimulate and regulate the function of the internal organs, promote the circulation of qi and blood, and maintain the balance of yin and yang of the body, so as to resist the invasion of external evil 3: “the patriarchal tendons bind the bones and benefit the organs.” It shows that the meridian tendons of the body can restrain the bones and flexion and extension joints and maintain the function of human movement coordination [33]. In the meridian syndrome differentiation of the body, the limb spasm of hemiplegic patients after stroke is in a state of limb spasm, the pathogenesis is the imbalance between yin and yang, the limb spasticity caused by “Yang slowness, yin urgency,” and the relative relaxation of the extensor muscle in the patient's limb relaxes the relative urgency of the flexor muscle so that the limbs show contracture and flexion. Acupuncture treatment can adjust yin and yang and restore the relative balance of muscle tension between extensor and flexor groups on the abnormal pattern of upper limb spasm; diarrhea has complementary deficiency and has a two-way regulatory effect [34]. The rehabilitation training alone has a short effect on the cerebral cortex, and the stimulation is not obvious. At the same time, although the cost of acupuncture alone is low, it cannot make hemiplegic patients establish a correct movement mode. The perception of the information of the movement pattern cannot be established, so a kind of therapy is often difficult to achieve the desired therapeutic effect. At present, the combination of multiple methods in the medical field is obvious for the recovery of motor function of hemiplegic patients. Traditional Chinese medicine acupuncture rehabilitation therapy eliminates fatigue, balances yin and yang through acupuncture treatment, and establishes a correct movement pattern in combination with rehabilitation exercise training, which can restore normal motor function [35].

The mechanisms of further recovery after central nervous system injury are brain plasticity and functional reorganization [36]. The former needs early repeated stimulation and directional induction to promote the opening of latent neural pathways, brain tissue reactive synaptic formation, peripheral nerve tissue axonal collateral sprouting, and so on. The latter includes the substitution of contralateral functional areas or ipsilateral peripheral tissues, which also requires repeated stimulation, motor learning, and functional training [37]. Therefore, the EMG biofeedback technique based on the principle of repetitive electrical stimulation is more and more used in clinical practice. Electromyographic biofeedback (EMG-BFB) therapy is a kind of biofeedback therapy [38, 39]. It is a microelectrical signal that is received, recorded, and displayed in the form of an image by a device to reflect muscle contraction that people do not normally feel and to provide intuitive visual and auditory feedback to patients through the observation screen. Through visual and auditory feedback information combined with instrument training, patients can carry out conscious self-repetitive training for some limbs with poor active activity and high muscle tension under the repeated stimulation and induction of the instrument. Therefore, EMG biofeedback therapy fully mobilizes the challenging psychology of patients and makes them cooperate in rehabilitation more actively and consciously, thus promoting the recovery of limb motor function and muscle spasm after stroke [40, 41]. Meta-analysis is a research method for systematic comprehensive evaluation and quantitative analysis of multiple independent research results with the same research purpose. This study included 5 RCTs, all of which met the diagnostic criteria, with a total of 750 stroke patients with hemiplegia. All are Chinese documents. Only two articles mentioned random assignment of study subjects, but the specific random assignment method was not reported. All literature reported blinded use, loss to follow-up, or delay. In this paper, the Fugl-Meyer motor function evaluation lower limb score, FCA walking function score, and lower limb Brunnstrom staging score were used to analyze the recovery of lower limb motor function in stroke patients with hemiplegia by acupuncture combined with rehabilitation training. The results of meta-analysis of this study show that hemiplegic patients after stroke who receive acupuncture combined with rehabilitation training can obtain better therapeutic effect and the motor function of the lower limbs of these patients is improved more obviously after treatment and its curative effect is better than that of conventional treatment. The limitations of this study are as follows: (1) the language is limited, only the published Chinese literature is searched, and the literature may be incomplete; (2) the level of domestic clinical evidence is low, there is a lack of high-quality and standardized RCT, and there may be selective deviation without strict randomization scheme and blind method; and (3) the number of included literature is small (only 5), and the included research information is limited, and the quality of methodology is not high. Therefore, the inclusion of the study may have some limitations, such as publication offset, language deviation, and clinical heterogeneity, which will inevitably affect the intensity of the results.

In conclusion, on the basis of routine treatment, acupuncture combined with rehabilitation training can restore the motor function of lower extremities in patients with acute stroke. At the same time, more high-quality randomized controlled studies are needed in the future.

## Figures and Tables

**Figure 1:** Forest plot of meta-analysis of the lower limb score based on Fugl-Meyer motor function assessment.

**Figure 2:** Forest plot of meta-analysis of the FCA walking function score.

**Figure 3:** Forest plot of meta-analysis of the lower limb Brunnstrom staging score.

**Table 1:** Basic characteristics of literature.

Include the literature	Year ofpublication	*N* (T/C)	Outcomeindex	Experimentaltime	Whether it is random or not	Whether it is blind or not	Jadad scoring
Fang Laiman	2021	52/48	①②③	1 month	No	No	1
Cai Xu	2015	100/100	①②③	4 months	No	No	0
Zhou Liangjun	2012	60/60	①②③	3 months	Yes	No	0
Hu Kehui	2013	32/30	①②③	1 month	Yes	No	0
Liu Chen	2018	37/37	①②③	1 month	Yes	No	1
Jingfuquan	2020	45/45	①②③	1 month	Yes	No	0
Wang Fengchuan	2010	80/80	①②③	4 months	No	No	0
Wu Ping	2015	45/45	①②③	4 months	Yes	No	1

## Data Availability

The datasets used and analyzed during the current study are available from the corresponding author upon reasonable request.
